# Design of Edge Computing Online Classroom Based on College English Teaching

**DOI:** 10.1155/2022/7068923

**Published:** 2022-06-14

**Authors:** Changhui Zhen, Kun Hu

**Affiliations:** ^1^Foreign Language Department, Bengbu Medical College, Bengbu 233000, China; ^2^Scientific Research Center, Bengbu Medical College, Bengbu 233000, China

## Abstract

This study expects to solve the network delay in college English online teaching, prevent disrupting the normal teaching order of college English classroom caused by network problems, increase college students' interest in learning English, and improve the time spent by college students in English learning. First, the study investigates and analyzes the current needs and situation of college English online learning and puts forward the improvement standards for college English online classroom. Second, the study applies edge computing (EC) technology to improve online teaching system and designs an online learning system for college specific English based on EC. Finally, the improvement effect is tested, and it is concluded that the effect of using EC to improve the online classroom system for college English is better than that of the unmodified online teaching system. The results reveal that the online classroom system for college English based on EC designed can effectively reduce the network delay of the traditional teaching system, ensure a high reliability, and increase the time for students to learn English, so it is helpful to improve the teaching quality. The results provide a new direction for applying emerging computer technology in online teaching in colleges and universities, a guarantee for improving college students' English level, and set an example for the relevant research in the future.

## 1. Introduction

With the popularization and rapid development of emerging network technology in China, online teaching has been widely used in various education industries. Due to the current environment, it is impossible to carry out offline teaching at some time, so it is necessary to develop applied online teaching systems. English has always been one of the most important subjects. In the process of English teaching, it is necessary to pay attention to the training of listening and speaking and make full use of computer equipment. At present, the online English teaching system has received extensive attention in the Corona Virus Disease 2019 (COVID-19) pandemic environment. Teachers can use the system to upload English courses, publish learning tasks, and conduct online teaching operations through the online teaching platform. Students can download course information and watch videos to learn. Fitria showed through research that online English learning systems had the potential to help lecturers and students more effectively in the teaching and learning process [1]. Rifiyanti found that online English learning was an important alternative to help to teach and learn under the COVID-19 pandemic. They considered using appropriate technology, quality, and teachers' ability of enhancing and encouraging learners to participate in the online learning environment [2]. Sun et al. developed an intelligent online English teaching system by combining artificial intelligence modules with knowledge recommendation. The system can help students improve the efficiency of English teaching according to their mastery of knowledge and personality. Meanwhile, it can help teachers improve their educational level and students' English scores and provide new ideas for the design and improvement of online English courses [3]. These studies suggest that the current research on the online English learning system focuses on analyzing its feasibility and function development, but few scholars pay attention to the operation efficiency of the system.

On the one hand, the current actual online teaching cannot reasonably apply and manage the teaching resources because of the limitation of various hardware facilities. On the other hand, the gradually popular cloud computing usually adopts centralized management, so it is unable to ensure the low delay and reliability of online classroom, or even causing some data security problems [4]. In this case, edge computing (EC) technology is introduced here to improve the current online teaching system. EC technology can provide closely integrated services using open platforms, combined with core capabilities of the network, computer, storage, and applications near objects or data sources. It can start the procedure on the edge to generate fast network service response and meet the basic needs of the industry in real-time business, application intelligence, and security and privacy protection. The edge computer is located between the physical subject and the industrial connection or above the physical subject. Compared with cloud computing, EC can perform data processing and analysis faster [5].

The application of EC technology in all walks of life has been studied by many domestic and foreign scholars. Wu and Song realized a content distribution framework for teaching monitoring videos through network, storage, and EC capabilities. Besides, they utilized Long Short-Term Memory (LSTM) to provide edge cache architecture and cache update strategy [6]. Sun proposed a system resource allocation method based on power iteration, which took the throughput of unloading process as the objective function and realized the optimal allocation of normal power through iterative optimization. Meanwhile, aiming at the problem of low energy efficiency and low resource utilization of edge servers, they constructed a heterogeneous network via edge servers to find the optimal strategy on the basis of ensuring Nash equilibrium [7]. Mehrabi et al. designed an optimized network-assisted adaptive solution, especially for mobile flows in multiaccess edge computing environments. They constructed a heuristic-based algorithm to minimize the demand for network parameter adjustment and reduce the network complexity. Besides, they investigated the performance of the solution against two popular client-based solutions, namely, buffer-based adaptation and rate-based adaption, and another network-aided solution [8]. Barthelemy et al. proposed an EC device, using computer vision and deep neural network to track real-time multimodal transport, while ensuring the privacy of citizens. Moreover, they developed an interoperable agnostic framework for collecting, storing, and accessing data from multiple sensors [9]. Wang et al. proposed a generation method of long-term prospect reference object library by existing large-scale monitoring vehicle object data set sharing. They also put forward a coding-oriented virtual foreground reference image generation method for object retrieval, to meet the requirements of low complexity and high-performance coding, which obtained satisfactory virtual foreground reference image effect and significantly reduced the delay [10]. Lv achieved a comprehensive technology combining multifield high-tech achievements to realize the human-computer interaction of Internet of Things (IoT) in a natural and intelligent way [11].

To sum up, at present, the research of EC technology is mainly concentrated in the fields of industrial production and traffic photography and seldom applied in education. This work innovatively uses EC technology to optimize the college English online teaching system, improve the online teaching system's stability, and help build a new teaching order and teaching model in the current epidemic environment. The integration of EC technology with IoT technology is utilized here to improve the online system of college English. Firstly, under the foundation of current teaching requirements analysis, EC is combined with the IoT technology for the online classroom to improve the network situation. The video stream frame filtering method is proposed to filter gibberish, and a corresponding algorithm is written for an online classroom system. Consequently, a teaching video transmission system with high real-time performance is obtained, which reduces the network delay and improves the reliability. The research results are of great significance to the education development in China and the promotion of online teaching technology.

## 2. Construction of New Online Classroom

### 2.1. Current Situation of Online English Teaching in Colleges and Universities

#### 2.1.1. IoT

The IoT technology was born in 1999 at Massachusetts Institute of Technology in the United States. It is an emerging information service architecture based on the Internet and radio frequency identification technology. This architecture aims to enable the information technology infrastructure to provide safe and reliable “goods” information through the Internet and to create an intelligent environment to identify and confirm “goods” to facilitate information exchange within the supply chain. IoT is developing rapidly today and is reforming human life mode, which permeates all aspects of human life, but also causes some problems. The IoT needs to verify the user before operation, providing an inherent leak difficult to solve from the technical perspective, and users can only be informed in advance in privacy policies [12, 13].

#### 2.1.2. Cloud Computing

Cloud computing is a service related to information technology, software, and the Internet, which can provide dynamically scalable and cheap computing services on demand through the network. It is also a computing model that provides dynamically scalable virtualized resources through the Internet in a service manner. Cloud computing has the following characteristics: large-scale, distributed, virtualization technology, high availability and scalability, and on-demand services. However, cloud computing still has the problems of low security, high cost, difficulty in governance, legal risks, lack of resources and expertise, immature technology, and high requirements for network quality. Cloud computing gathers all data on the edge of the network and processes data on the main server. Cloud architecture is famous because most devices, such as smartphones, are near the edge without sufficient storage capacity and computing power, which cannot process or analyze the collected data. Although people can use WiFi or other high-speed networks on most devices, their hardware capabilities remain limited. Therefore, ordinary devices are inadequate for data processing or analysis [14–16].  Figure 1 illustrates the architecture of the cloud platform.

Generally accepted cloud architecture usually consists of three layers: the infrastructure layer, the platform layer, and the software service layer. The corresponding names are Infrastructure as a service (IaaS), Platform as a Service (PaaS), and Software as a Service (SaaS). IaaS mainly includes computer servers, communication devices, and storage devices to provide users with information technology infrastructure services such as computing capacity, storage capacity, or on-demand network capacity, which are provided at the infrastructure level. The core of IaaS's mature application lies in virtualization technology. Through virtualization technology, it can virtualize all kinds of computing devices into computing resources in the virtual resource pool, virtualize storage devices into storage resources in the virtual resource pool, and virtualize network devices into network resources in the virtual resource pool. When users order these resources, the data center manager directly packages the ordered shares and provides them to users, thus realizing IaaS.

#### 2.1.3. College English

College English is a compulsory public basic course for most non-English majors. It mainly cultivates college students' foreign language ability, humanistic quality, and cross-cultural communication ability. College English teaching objectives can be divided into three levels: foundation, improvement, and development. College English teaching can adopt task-based, cooperative, project-based, inquiry, and other teaching methods. *The College English Teaching Guide* (2020 edition) points out that college English should give full play to the important role of modern information technology in English teaching and vigorously promote the deep integration of modern information technology and English teaching.

According to *the Guide*, college English teachers should make full use of network teaching platform, make rational use of information technology elements, innovate, and practice online teaching mode and online and offline mixed teaching mode. Colleges and universities should make full use of information technology and actively create a diversified teaching and learning environment. *The Guide* pays special attention to promoting the modernization of college English teaching means. The construction of a new education and teaching model based on information technology has become a national strategy [17].

#### 2.1.4. Online English Teaching

During the novel coronavirus pneumonia epidemic prevention and control, online teaching provided an important opportunity to consolidate English teaching concept and innovate teaching methods and means. The development of Internet plus, intelligence + technology online, and offline education has become an important development direction of higher education in China and the world. Our English online teaching system mostly adopts cloud computing technology and online teaching platforms in colleges and universities and relies on courseware made by teachers and a few application systems. Although online teaching has been achieved, there is a serious shortage of teaching resources. The new educational intelligent cloud classroom today can support online real-time learning or lecturer video playback. In particular, online real-time learning requires good network conditions and cloud processors with extremely large memory space [18, 19].

The test of the learning module of online real-time classroom proves frequent network delays or lags. Moreover, when more than half of the students watch the learning videos recorded by the lecturers synchronously, the buffer time of the videos will be greatly prolonged. This is because the online teaching student terminals frequently send requests and uploads or downloads data to the cloud server, which gradually accumulates the amount of data needed to be processed by the cloud server. The excessive mass of data will reduce processing speed. Besides, these behaviours will occupy a large network bandwidth, further reducing the speed of data transmission, and seriously limiting functions of the cloud computing system.

### 2.2. EC Technology

EC is a kind of cloud computing technology. Since it processes data near the data source rather than in the external data center or cloud, it can reduce the network delay time. Besides, it requires a low cost, so users spend less on data management solutions of local equipment than on cloud and data center networks. As the number of IoT devices increases, data generation continues to increase at a record rate. Correspondingly, the network bandwidth becomes limited, making the cloud overwhelmed and causing greater data bottlenecks. EC has higher application running efficiency, because with the decrease of lag the application can run faster and more efficiently. Since MEC (mobile edge computing) technology has an independent server and strong computing and storage capabilities, with the server extremely close to the network terminal equipment on the physical layer, it also greatly improves the user's service experience. Moreover, through EC, the network model can be adjusted according to individual needs based on constant learning, bringing personalized interactive experience. Furthermore, EC is concentrated, effectively avoiding personal privacy leakage [20–22].  Figure 2 reveals the architecture of the EC system.

The cloud edge nodes in Figure 2 contain SaaS, PaaS, and IaaS. SaaS is a software application mode to provide software services through the Internet. In this mode, users do not need to spend much investment on the construction of hardware, software, and development teams. They only need to pay a certain rental fee to enjoy the related services through the Internet and enjoy the maintenance of the whole system provided by the manufacturer. From the perspective of “hardware + operating system/Development Tools +  application software” in traditional computer architecture, the platform layer of cloud computing should provide functions similar to the operating system and development tools. Similarly, PaaS aims to provide users with a supporting platform for developing, running, and operating application software through the Internet. Just as in the personal computer software development mode, programmers may use development tools to develop and deploy application software on a computer equipped with windows or Linux operating system.

Users are trying to utilize IoT devices to optimize the network, hoping to locate the processing function at the edge of the network and accomplish real-time data processing and analysis. The EC system does not need to return data to the server, which reduces network delay and improves processing performance. In addition, EC is conducive to optimize the data-driven function of the network by collecting, analyzing, and processing data close to the end user [23].  Table 1 demonstrates the advantages of EC.

### 2.3. Video Live Broadcast and Recording Technology via EC Technology

#### 2.3.1. EC Video Live Broadcast Framework

EC technology can transfer cloud computing to the edge side of the network, to meet the real-time requirements of the network, providing more efficient data processing, more intelligent application functions, and more guaranteed data security. The network video live broadcast and recording system based on EC technology can transfer the main processing steps of video information to EC devices instead of transmitting data to the cloud for processing. Besides, the EC video live broadcast framework can remove background noise and redundant data information in the image and make better judgment and decision on image content. When the complex processing is transferred to the EC center for calculation and storage, the requirements for bandwidth and network speed decrease. Moreover, since the EC platform has the function of user information security protection and early warning, it can better protect the security and privacy of users. The edge side of the video live broadcast and recording framework uses cameras for initial video data collection. When the edge side transmits data to its edge cloud server, it also manages and schedules the front edge devices in all paths, thus monitoring the information security and transmission capacity of the front edge devices. The front-end edge device and server will preprocess the received data information and filter out the unnecessary data information, to reduce the space occupied by video information and improve the overall efficiency of video information storage. This also provides a solution to the insufficient storage space in the EC system and the network delay problem, alleviating the network pressure and eliminating the security problem caused by network bandwidth [24, 25].

In general, it is necessary to connect numerous front edge devices and server vectors for the bidirectional information transmission. Besides, the data transmission between front edge devices and servers and between the servers and the cloud centers must adopt the bidirectional transmission technology. This system includes hardware layer and software layer. The hardware layer needs to use the computing hardware unit, wireless communication module, and video terminal equipment to communicate with the outside. The software layer involves some image processing algorithms. The preprocessing steps are completed by the front edge device, while information fusion and state estimation are operated by the server. Finally, the result report is transmitted to the cloud center, and the service management is carried out by the cloud center [26].  Figure 3 presents the EC video system.

Figure 4 provides the video analysis process, including four steps.

#### 2.3.2. Video Data Acquisition

Video stream is used to describe the bidirectional transmission of data. If a video stream becomes stable and continuous after the processing of network and video compression algorithm, it is called a coding stream. The compression coding algorithm used here is H. 264. The original unprocessed video stream is called YUV stream (Y), which is almost used for the compression of all the transmission streams in the network. When the data stream reaches the terminal, it will be decoded and converted to the decoded video stream called RGB [27, 28]. The YUV stream structure is shown in Figure 5.  Table 2 shows the structure of H. 264 packets.

In Table 2, NALU represents a set of NALU header information corresponding to video coding and original byte sequence payload; SPS signifies the sequence parameter set; Iframe represents the intracoded frame; PFrame refers to the forward prediction coding frame; BFrame represents bidirectional prediction interpolation coding frame.

#### 2.3.3. Transfer Protocol (TP)

The categories of video TP are mainly Hypertext Transfer Protocol (HTTP) and Real-time Transport Protocol (RTP). RTP is divided into Real-Time Controlling Protocol (RTCP) and Real-Time Streaming Protocol (RTSP). RTSP is adopted here because it is suitable for transmitting large files [29, 30].

The transmission process of RTSP is composed of the following sections. (a) The user terminal device is connected with the server, which communicates in the form of command description characters. (b) After receiving the communication command, the server returns a series of corresponding characters as a response. (c) After receiving the response string sent by the server, the user terminal establishes the corresponding commands for the individual flow in the response content according to the response type, to inform the server with the actual port collecting the data. (d) After the establishment of the basic connection condition, the user terminal transmits the corresponding request to guide the server to run, so the server will send the media flow data packet required by the client terminal. In this step, the user terminal can send different requests to adjust the process of server running. (e) This step corresponds to the end stage of the communication between the client terminal and the server. In this stage, the client terminal needs to send a request to guide the end of the whole communication.  Figure 6 indicates the complete RTSP running process.

#### 2.3.4. Video Frame Filtering Algorithm

The effect of video frame filtering is to cut the video stream according to time *T*, to attain many video frame sequences with different contents and form a group. Then, the system identifies the video frame sequences to find the required part. Frames per Second (FPS) represents the number of frames transmitted in each second or the number of RGB format images transmitted in each second, and FPS is related to the fluency of the display picture. The higher the FPS is, the smoother the picture is. 24 FPS is generally used currently. Denote the result amount included by the main frame *i* in the total video stream *S* by *O*_*i*_, the broadband transmission experiment by *D*_*e*_, the complexity of the algorithm by *O*(*T* ∗ *X*), the frame length by *T*, and FPS by *F* [31].

### 2.4. Optimization of the EC Video System Based on Cooperative Computing

#### 2.4.1. Cooperative Computing Optimization

Collaborative computing contains two core parts: symmetric processing and parallel processing. However, due to the delay of network response, the current technology cannot complete the symmetric processing. Therefore, the parallel processing mode is adopted here; that is, multiple different tasks are processed simultaneously. Collaborative computing is a kind of optimization algorithm, which uses edge server to allocate data processing tasks and sends the task to the terminal with computing components, such as intelligent cameras and intelligent sensors. This method can greatly improve the speed of data processing and reduce the delay and system load [32].  Figure 7 presents the comparison of allocation schemes between noncooperative and cooperative computing under EC.

#### 2.4.2. Optimization of the Data Processing Allocation Scheme by Cooperative Computing

The data to be processed is distinguished by complexity, as shown in

(1) $$\begin{array}{c} W=\sum_{i=1}^{n}K_{n}w_{n}\left(w_{1}<w_{2}<...<w_{n}\right). \end{array}$$

In (1), *W* represents the total workload of data to be processed; *k*_*n*_*w*_*n*_ denotes the workload of a single data with difficulty *n*; *K*_*n*_ stands for the processing times required for data with difficulty *n*; *v* represents the total workload of processing data with difficulty *n* [33].

It is necessary to select the location for the placement of EC center and user terminal. The first following equation describes the data on the location of EC center, and the second following equation represents the location of user terminal:

(2) $$\begin{array}{c} E_{0}=\left(d_{0}=0,B_{0}=0,c_{0},v_{0}\right), \end{array}$$

(3) $$\begin{array}{c} l_{j}=\left(d_{j},B_{j},c_{j},v_{j}\right). \end{array}$$

Among (2) and (3), *d* represents the linear distance between the terminal and the server, while *B* denotes the data transmission bandwidth. In addition, *c* refers to the data processing capacity, and *v* signifies the data processing speed.

Mark *X* as a reasonable allocation scheme, and the matrix model for data processing can be expressed as

(4) $$\begin{array}{c} T_{\text{total}}=\arg\;\min w^{T}X\bar{V}+2d^{T}V, \end{array}$$

where *T*_total_ represents the sum of time required for data processing and arg min denotes the corresponding value of *X* when *T*_total_ is the smallest. Then, set the server's initial processing capacity to *c*_0_, the initial processing speed to *v*_*o*_, and the light speed is *s*. Then, there are

(5) $$\begin{array}{c} c={\left(c_{0},c_{1},\ldots ,c_{m}\right)}^{T}, \end{array}$$

(6) $$\begin{array}{c} d={\left(d_{0},d_{1},\ldots ,d_{m}\right)}^{T}, \end{array}$$

(7) $$\begin{array}{c} V={\left(\frac{1}{s},\frac{1}{s},\frac{1}{s},\ldots ,\frac{1}{s}\right)}_{1\times \left(n+1\right)}^{T}, \end{array}$$

(8) $$\begin{array}{c} \bar{k}={\left(K_{1},K_{2},K_{3},\ldots ,K_{n}\right)}_{1\times n}^{T}, \end{array}$$

(9) $$\begin{array}{c} B={\left(0,\frac{1}{B_{1}},\frac{1}{B_{2}},\ldots ,\frac{1}{B_{m}}\right)}_{1\times \left(n+1\right)}^{T}, \end{array}$$

(10) $$\begin{array}{c} \bar{V}={\left(\frac{1}{v_{0}},\frac{1}{v_{1}},\frac{1}{v_{2}},\ldots ,\frac{1}{v_{m}}\right)}_{1\times \left(n+1\right)}^{T}, \end{array}$$

where $\bar{k}$ indicates the average data processing times; $\bar{V}$ represents the average data processing speed. Define a unit column vector *I* of 1 × (*n* + 1) and define the matrix *X* as the optimal allocation strategy of function arg min, and the matrix *X* is *n* × (*m* + 1)-dimensional matrix of the content adjusted with the strategy.

According to the complexity of data processing and matrix *X*, the total processing quantity *W* is quantified into three parts. Denote the processing quantity of the server by *W*_Edge_, the processing quantity of the terminal by *W*_devices_, and the processing quantity of the *j*th terminal by *W*_*j*devicese_, which can be written as

(11) $$\begin{array}{c} W_{\text{Edge}}=\sum_{i=1}^{n}w_{i}k_{i0}, \end{array}$$

(12) $$\begin{array}{c} W_{j\text{ devices}}=\sum_{i=1}^{n}w_{i}k_{ij}, \end{array}$$

(13) $$\begin{array}{c} W_{\text{devices}}=\sum_{i=1}^{n}W_{j\text{ device}}. \end{array}$$

### 2.5. Design of Experiments

#### 2.5.1. Experiment for the Video Transmission Effect

The processing results of 10 frames in the same time period of two video streams *S*1 and *S*2 are selected for the experiment, which are processed by video filtering technology as the following steps. (a) Calculate the average recognition result O*i*, *s* of the video stream S within the *T* period, and perform frame filtering for the video stream path with large *Os*. Repeat the operation until the number of target recognitions is not less than the average recognition result. (b) Select and reserve the frame with changes in *O*_*i*_, *s*. (c) Sort the frames obtained in the previous step according to the size of *O*_*i*_, *s*, and generate the obtained result into a sequence group. The filtering of video frames with a large number of target recognitions is stopped first.

Four kinds of data resolution are selected for network delay comparison experiment, namely, 320P, 480P, 720P, and 1080P.

The actual availability of broadband is detected when the bandwidth is 5 Mbps, 10 Mbps, 15 Mbps, 20 Mbps, and 25 Mbps, respectively.

#### 2.5.2. Evaluation of the Practical Application Effect of the System

The textbook of New Horizon College English is taken as an example for the experiments to verify the practical application effect of the online English learning system proposed here. First, the teacher randomly selects a unit of content in the textbook, makes network courseware, and initiates a collective video to start online teaching. The timing starts until the teacher finishes explaining all the contents. In this process, the times of video jamming and blurring are recorded and compared with the system without EC optimization.

## 3. Experiment of the Effect of EC Online Classroom

### 3.1. Improvement Effect of Video Stream Filtering on Network Delay

Figure 8 illustrates the target recognition number of the video streams by the filtering system, and Figure 9 demonstrates the average video processing delay.

As shown in Figures 8 and 9, these sequence groups of video frames are formed after filtering: [2, 6], [5, 7], [0, 2], and [2, 9]. Moreover, the whole process goes smoothly, and there is no error due to the algorithm. After loading the network frame filtering algorithm, the required time for data analysis and processing is significantly reduced. The data after frame filtering contains more effective information, thereby reducing the analysis time, reducing the average delay, and increasing real-time performance. When the image resolution reaches 720P, the average frame processing delay is reduced from 43 milliseconds to 31 milliseconds, decreasing by 12 milliseconds. When the resolution is 1080, the average frame processing delay decreases from 58 milliseconds to 41 milliseconds, down by 17 milliseconds. This shows that the higher the resolution is, the more the average transmission delay decreases after frame filtering. The reason for this phenomenon is that the increase in resolution leads to the increase in the definition of video frames, which can improve the performance of the filtering algorithm.

### 3.2. Improvement Effect of Video Stream Filtering on Network Bandwidth Utilization

Figure 10 reveals the network utilization at different network bandwidths.

When the network bandwidth is between 5 Mbps and 5 Mbps, the frame filtering algorithm is used to filter the frames under different network bandwidths, which ensures real-time video data transmission. After video frame filtering algorithm processing, the filtered FPS is mainly distributed in the range of 15 to 22. The edge node task scheduling optimization algorithm improves network utilization compared with the ordinary video frame filtering algorithm. Under good network bandwidth, the node task scheduling optimization can be efficiently and effectively executed, so network utilization can be maintained at more than 99%. When the network bandwidth is poor, the network utilization rate remains above 80%.

### 3.3. The Evaluation Results of the Practical Application Effect of the System

Figure 11 presents the test results of total course time and video lag times when using the optimized system reported here and the original system for teaching.

As shown in Figure 11, when using the unoptimized system, the whole course takes 46 minutes; when using the optimized system, the whole course takes 29 minutes, which is 37% shorter than the original system. Besides, the number of video jams and blurs is 54.5% and 66.7% less than the original system, respectively. The results prove the advantages of the optimized system in video transmission efficiency and image processing.

## 4. Conclusions

The original college English online learning system is improved based on EC and IoT technology. Firstly, the current online learning needs and status of college English are analyzed. Then, the advantages of EC and IoT technology for online teaching system improvement are analyzed. Subsequently, an online learning system for college English based on EC technology is designed. Finally, the improvement effect is tested, and it is concluded that the EC technology can effectively improve the online learning system. The results demonstrate that the online learning model of college English based on EC can effectively reduce the network delay of general technology, ensure high reliability, and solve the current network problems of online teaching. Thus, an excellent online teaching system can be obtained, which is conducive to improve the learning efficiency of college students' English.

This work optimizes the online English learning system using EC, which dramatically improves the speed and stability of network data transmission. However, the function design of the system in practical teaching application and the maintenance of students' classroom discipline were not comprehensively considered. The future study will combine the Deep Learning technology with the online English learning system and refine the system to improve the practicability and help lecturers monitor students' daily attendance, maintain classroom discipline, and improve the online English classroom mode.

## Figures and Tables

**Figure 1:** Architecture of the cloud platform.

**Figure 2:** Architecture of the EC system.

**Figure 3:** EC video system.

**Figure 4:** Video analysis process.

**Figure 5:** Structure of the YUV stream.

**Figure 6:** Complete RTSP running process.

**Figure 7:** Comparison of allocation schemes between noncooperative and cooperative computing under EC.

**Figure 8:** Target recognition number of the video streams by the filtering system.

**Figure 9:** Average video processing delay.

**Figure 10:** Network utilization at different network bandwidths.

**Figure 11:** Evaluation results of the practical application of the system.

**Table 1:** Advantages of EC.

No.	Merit	Specific advantage
1	Network speed	The most significant superiority of EC is the speediness, which can reduce network delay. With EC, the IoT device will process data in the edge data center or locally. Therefore, data need not be transmitted back to the central server.

2	Network security	If all data is transmitted back to the main server, the operation process and data are vulnerable. A Distributed Denial of Service (DDoS) attack is sufficient to disrupt the entire business process. EC will allocate data processing between different data centers and devices. Therefore, the network will be difficult to be attacked by DDoS attacks, which will also increase the total area of attacks. Therefore, hackers cannot affect the entire network by attacking a device. If the data is stored and analyzed locally, the security team can easily monitor them. This will also help users overcome privacy laws.

3	Expandability	EC can easily extend the infrastructure and extend the edge network by buying devices with sufficient computing power. Users do not need to build their own private or centralized data centers for their data needs. On the contrary, they can extend edge networks by combining EC with hosting services at a lower cost.

4	Reliability	Compared with cloud computing, EC provides better reliability. All edge data centers and IoT devices are located near users in the EC system. Therefore, the network is less like being interrupted. If the user's edge center is unavailable, the IoT device will automatically process the request, and the IoT device can handle most functions independently. Each traditional data center also has some limitations on the amount of data that can be transmitted.

**Table 2:** Structure of H.264 packets.

SPS	NALU
SPS	
Iframe	
Iframe	
PFrame	
BFrame	
BFrame	
PFrame	
PFrame	

## Data Availability

All data are fully available without restriction.
